This article has been retracted.

# Chinese Herb Jiedu Huayu Granules Inhibiting Immune and Inflammatory Response of Rats with Acute Liver Failure by Regulating the NF-*κ*B Signaling Pathway

**DOI:** 10.1155/2022/4479885

**Published:** 2022-05-11

**Authors:** Wenjie Bai, Qinglan Shi, Jinyu Wu, Kejing Wang, Yueqiao Chen, Xiaocong Ma, Dewen Mao

**Affiliations:** ^1^Foreign Language Department, Guangxi University of Chinese Medicine, Nanning, China; ^2^Department of Liver Diseases, The First Affiliated Hospital of Guangxi University of Chinese Medicine, Nanning, China; ^3^Hepatobiliary Surgical Department, Ruikang Hospital Affiliated to Guangxi University of Chinese Medicine, Nanning, China

## Abstract

**Objective:**

To research the influence of Chinese medicine Jiedu Huayu granules (JDHY) on the immune response and inflammatory response of rats with acute liver failure (ALF) and investigate its related mechanism.

**Methods:**

Rats were randomly divided into 4 groups: control group (*n* = 6) were injected with the same amount of normal saline; ALF group (*n* = 10) were injected intraperitoneally with D-GaIN (700 mg/kg) and LPS (10 *μ*g/kg); ALF+JDHY group (*n* = 10) were given JDHY 57.55 g/kg/d by gavage for 7 days and injected intraperitoneally with D-GaIN/LPS after the last dose; and ALF+BAY group (*n* = 10) were given BAY 10 mg/kg/d by gavage for 7 days and injected intraperitoneally with D-GaIN/LPS after the last dose. Changes in liver function and coagulation function were examined in rat serum; the pathological varieties of liver tissues were verified by HE staining; immunohistochemistry was utilized to determine the ratio of PCNA and F4/80 in liver tissues; the flow cytometry was applied to determine the ratio of CD4+/CD8+ cells in peripheral blood mononuclear cells (PBMCs); ELISA and qRT-PCR were utilized to check the level of IL-10, IL-6, IL-13, IL-1*β*, TNF-*α*, IFN-*γ*, and CD163 in serum and liver cells. Western blot was adopted to check the expression of apoptotic protein and expression and NF-*κ*B pathway-related protein expression.

**Results:**

JDHY and BAY could decline the expression of AST, ALT, ALP, and TBiL in ALF rat serum significantly (*P* < 0.01), increase PTA and PLT (*P* < 0.01), and mitigate liver tissue damage. Besides, JDHY and BAY could reduce the apoptosis and improve the proliferation of the liver cells in rats with ALF; meanwhile, the ratio of CD4+ cells and F4/80 cells was reduced while CD8+ cells were increased (*P* < 0.01). Further, JDHY and BAY could reduce the level of IFN-*γ*, IL-6, IL-1*β*, and TNF-*α* while increasing the level of IL-10 and IL-13 (*P* < 0.01). Additionally, the expression of sCD163 in serum and CD163 expression in liver tissues increased (*P* < 0.01). The result of western blot confirmed that JDHY could inhibit the phosphorylated expression of NF-*κ*B, IK*βα*, and IKK*β* in the ALF rat tissues.

**Conclusions:**

JDHY can upregulate the level of CD163/sCD163 by the NF-*κ*B signaling pathway, thereby regulating immune response, inhibiting inflammatory response, and ultimately improving ALF in the rats.

## 1. Introduction

Acute liver failure (ALF), mainly created by a series of liver diseases, is a liver syndrome that remains to have a great mortality. The mortality of ALF reached 60%-80% [1, 2]. The patients with ALF exhibit the features of a proinflammatory state of local liver inflammation, vascular endothelial dysfunction, and systemic inflammatory response syndrome (SIRS) [3]. All these features promote the development of multiple organ failure [3]. Systemic inflammation is its main feature, and its adverse prognosis is closely related to the intensification of systemic inflammatory response known as cytokine storm. Imbalance of immune function is an important pathogenesis of ALF [4]. Macrophages have multiphenotypic and multifunctional effect in liver regeneration. The defense of host against various protozoa, bacteria, and viruses is induced by classically activated macrophages (M1 macrophages), and proinflammatory cytokines, such as interleukin- (IL-) 6 and tumor necrosis factor *α* (TNF-*α*), are released [5, 6]. M2 macrophages are exposed in CD163. M2 macrophages have anti-inflammatory effects. Specifically, immunomodulatory mediators (such as IL-10) released by M2 macrophages can regulate inflammatory response and accelerate tissue remodeling [7].

In recent years, with 30% of ALF patients undergoing liver transplantation, the survival rate has improved [8]. However, the prognosis of patients is unsatisfactory due to the rarity and severity of ALF [8]. Traditional Chinese medicine has a certain history in dealing with liver failure, and the curative effect is good. Traditional Chinese medicine can protect hepatocytes from multiple targets, aspects, and levels. Chinese medicine Jiedu Huayu granules (JDHY) are a clinical prescription summarized according to toxic pathogen theory. JDHY is made up of red peony root, Artemisia capillaris, Hedyotis diffusa, rhubarb, radix curcumae, and Acorus calamus, including the effects of improving blood circulation for clearing away blood stasis, removing heat and toxic substances, normalizing the gallbladder to cure jaundice, and eliminating phlegm to wake up the mind. Further, the approval document of hospital preparations has been obtained (preparation batch number Z20110004) [9]. JDHY has been one of the most commonly used traditional Chinese medicine prescriptions for the treatment of chronic liver failure for more than twenty years. It can often achieve good curative effect, but its mechanism is not clear. It is confirmed that JDHY can interfere with the releasing of inflammatory factor through the I*κ*B/NF-*κ*B signaling pathway [10, 11]. Additional, early experiments have verified that JDHY can ameliorate the synthesis, secretion, and detoxification function of the liver in liver failure rats, reduce hepatic necrosis, prevent hepatocyte mitochondria, inhibit hepatocyte apoptosis, and improve the survival of rats [12, 13]. However, the relevance of JDHY and immunity in ALF rats remains unknown. Therefore, in this study, D-GaIN/LPS was utilized to induce the ALF rat model [14], and then, the effects of JDHY on immunity and inflammation in ALF rats were observed. All these were aimed at offering in-depth theoretical support to validate the effectiveness of JDHY in clinical medication.

## 2. Materials and Methods

### 2.1. Experimental Animal

Hunan SJA Laboratory Animal Co., Ltd. (China) offered 36 healthy SPF SD male rats (age: 6-8 weeks; weight: 170-230 g). These rats were housed in temperature-controlled environment (22°C) with a relative humidity of 50% as well as light/dark cycles for 12 h with ad libitum diet. This experiment was supported through the Guangxi University of Chinese Medicine Institutional Animal Ethical and Welfare Committee (DW20210310-041).

### 2.2. Establishment and Treatment of the Model of Rats with Acute Liver Failure

In total, 36 Sprague-Dawley (SD) rats weighing 170-230 g (6-8 weeks old, *n* = 18 females, *n* = 18 males) were nourished in a clean animal laboratory with a humidity of 55%–65% at 20–25°C. After 7 days, rats were randomly divided into 4 groups: ALF group (*n* = 10): D-GaIN (700 mg/kg) and LPS (10 *μ*g/kg) (Sigma, USA) were injected intraperitoneally [14]; ALF+JDHY group (*n* = 10): JDHY was fed through consecutive 7-day gavage at 57.55 g/kg/d and D-GaIN/LPS was injected intraperitoneally 72 h at after the last dose [15]; ALF+BAY group (*n* = 10): BAY was fed through consecutive 7-day gavage at 10 mg/kg/d and D-GaIN/LPS was injected intraperitoneally after the last dose; and control group (*n* = 6): rats were given an infusion of normal saline in a volume equal. After 6 h, rats were anesthetized with 30 mg/kg pentobarbital sodium, and then, the left lobe of the liver was picked from the abdominal cavity. About 0.2 g of tissue at the identical location was cut, and venous blood was collected from inferior vena cava under sterile conditions.

### 2.3. Biochemical Analysis

The serum of rats was collected. Corresponding biochemical kits (Nanjing Jiancheng Bioengineering Institute, China) were adopted to detect the level of total bilirubin (TBiL), alanine aminotransferase (ALT), aspartate aminotransferase (AST), and alanine aminotransferase (ALP) in the serum in each group.

The Coulter counter was used to count platelet (PLT). The prothrombin time of peripheral blood thrombin (PT) was measured through the prothrombin test kit (Nanjing Jiancheng Bioengineering Institute, China). And prothrombin activity (PTA) was calculated.

### 2.4. Histopathologic Analysis by Hematoxylin-Eosin (HE) Staining

HE staining steps referred to Li et al. [14]. Liver tissues were selected from rats at the identical sites of the model and normal groups to observe the morphological changes. After the 24 h fixation in 10% neutral formalin solution, the liver tissues were dehydrated with graded ethanol, permeabilized with xylene, embedded in paraffin, and sliced to 5 *μ*m continuously. Sections were deparaffinized with xylene after being dried at 60°C and dyed with hematoxylin and eosin after gradient alcohol hydration. Harris hematoxylin was added to stain for 7 min. The sections were rinsed with tap water for 1 min in 1% dilute. Hydrochloric acid was used for a few seconds, and they were washed with distilled water for 10 min to turn blue when they were exposed to ammonia in several seconds. Next, the sections were rinsed using tap water for 1 min and distilled with water 3 times and then stained with 1% eosin for 3 min. Also, they were rinsed with distilled water for 10 min and added with ethanol before being mounted in neutral balsam. Finally, the tissues were observed and photographed under a 400x optical electron microscope.

### 2.5. Flow Cytometry

Peripheral blood mononuclear cells (PBMCs) in whole blood of rats in each group were isolated using PBMCs' isolation kit (Solarbio, China). After these PBMCs were washed once, CD3, CD4, and CD8 antibodies (BD, America) were added to stain for 30 minutes at 4°C. And then moderate fluorescently labeled secondary antibodies were added to incubate at 4°C for 30 min. CD3+CD8+ T cells and CD3+CD4+ T cells in peripheral blood of rats in each group were tested through a flow cytometer, and the ratio of CD4+/CD8+ was calculated.

### 2.6. Immunohistochemistry

Immunohistochemistry steps referred to Li et al. [14]. The sections with the size of 4 *μ*m were obtained from the paraffin-embedded liver tissues of rats. Primary antibodies PCNA and F4/80 (1 : 500, Santa Cruz Biotechnology, USA) were put for incubation overnight at 4°C. Then, HRP-conjugated goat anti-mouse antibody was added for subsequent incubation. Immunohistochemistry was visualized through the diaminobenzidine (DAB) kit. The sections of liver tissues of rats were viewed at 200x magnifying glass. The staining intensity of PCNA and F4/80 in six random fields of per section was analyzed through imageproplus6.0. The rate of PCNA- and F4/80-positive cells was analyzed quantitatively. Each sample was analyzed in triplicate.

### 2.7. ELISA

According to the instruction of the ELISA kit (eBiosciences, San Diego, CA, USA), the amount of IL-10, IL-13, IL-6, IL-1*β*, IFN-*γ*, TNF-*α*, and sCD163 in serum of rats was measured.

### 2.8. qRT-PCR

Total RNA in liver tissues was obtained by the Trizol. And the reverse transcription kit (Takara, Japan) was utilized to synthesize cDNA. The cDNA was amplified according to the instruction of the PCR kit (Takara, Japan). The dissolution curve and amplification curve were obtained at the end of amplification. Then, quantitative analysis was conducted. With GAPDH as an internal reference, relative gene expression was calculated through the 2 − ΔΔCt method. The primers and sequences are shown in Table 1.

### 2.9. Western Blot

Total proteins were obtained after tissue lysate was added into rat liver tissues in each group. The BCA assay was applied to measure the content of total proteins. Equal amounts of proteins (20 *μ*g) were separated by electrophoresis. Then, these proteins were shifted to PVDF membranes. Subsequently, 5% nonfat dry milk was added, and the membranes were sealed for 1 h at 37°C. Then, the membranes were incubated with primary antibodies Bax, cleaved caspase-3, Bcl-2, CD63, IKK*β*, p-IKK*β*, I*κ*B*α*, p-I*κ*B*α*, NF-*κ*B, p-NF-*κ*B, and *β*-actin (Abcam, UK) overnight at 4°C. Further, the washed membranes were incubated with the secondary antibody IgG-HRP (1 : 5000) for 1 h at 37°C. After being washed, the membranes were observed by enhanced chemiluminescence (ECL) with the *β*-actin working as an internal reference. Images were obtained after the film by a transmission scanner, and the gray values of the electrophoretic bands were analyzed with ImageJ. Independent experiments were repeated for three times.

### 2.10. Statistical Analysis

All experimental data was analyzed through SPSS 22.0 software. Mean ± standard deviation (mean ± SD) was utilized to express the measurement data. Student's *t*-test or one-way analysis of variance (ANOVA) was applied to compare the discrepancies between two groups or among over two groups. *P* < 0.05 was thought to be statistically significant.

## 3. Results

### 3.1. JDHY Can Improve Liver Damage in Rats with Acute Liver Failure

The biochemical indicators in the serum were first examined. And the results indicated that, in the ALF group, the level of ALT, AST, ALP, and TBiL in the rat serum was higher compared with that in the control group (Figures 1(a)–1(d)). Meanwhile, compared with the control group, the level of plasma thromboplastin antecedent and platelet was notably downregulated in the rat serum in the ALF group (Figures 1(e) and 1(f)). After liver tissues in rats were further stained, the ALF group showed obvious pathological changes, including necrosis of liver cells, destruction of the lobular structure of the liver, infiltration of inflammatory cells in the lobules and periportal areas, and blood stasis in the sinusoids (Figure 1(g)).

However, in the serum of ALF rats pretreated with the JDHY or NF-*κ*B inhibitor BAY, the level of AST, ALT, ALP, and TBiL was upregulated significantly (Figures 1(a)–1(f)). The result of the histopathological test also indicated that inflammatory cell infiltration was significantly declined, and the lobular architecture in rat liver tissue was restored (Figure 1(g)). These results showed that JDHY or inhibition of the NF-*κ*B signaling pathway could reduce liver damage in ALF rats.

### 3.2. JDHY Can Decline Liver Apoptosis in Rats with Acute Liver Failure

The effect of JDHY on liver apoptosis in ALF rats was further evaluated. According to the result of western blot, compared with the control group, apoptotic protein Bax expression and cleaved caspase-3 expression were notably increased in the liver tissues of the ALF group, and Bcl-2 expression was significantly declined, while after adding JDHY and BAY, both Bax and cleaved caspase-3 expression were significantly declined in the liver tissues of ALF rats and Bcl-2 protein expression was significantly upregulated (Figure 2(a)). Immunohistochemical results also indicated that the positive expression of PCNA in liver tissues of the ALF group was markedly lower compared with that of the control group. Through the addition of JDHY and BAY, the level of PCNA was increased (Figure 2(b)). These results suggested that JDHY could reduce apoptosis of liver cells and promote their proliferation in ALF rats.

### 3.3. JDHY Can Restore Immunomodulation and Reduce Inflammatory Response in Rats with Acute Liver Failure

The effect of JDHY on immunomodulation in ALF rats was further analyzed. Flow cytometry result indicated that, compared with the control group, CD4+ T cells in PBMCs were significantly reduced, whereas CD8+ T cells notably increased, and the ratio of CD4+/CD8+ was declined notably in the ALF group, indicating an immune dysfunction in rats with liver failure. However, after ALF rats were pretreated with JDHY or BAY, CD4+ T cells were significantly upregulated, whereas CD8+ T cells were notably reduced, and the ratio of CD4+/CD8+ was upregulated (Figures 3(a) and 3(b)).

The expression of the macrophage-associated marker (F4/80) was further examined. The result indicated that F4/80 expression in ALF rats' liver tissues was higher compared with that in the control group, where in the ALF+JDHY group and ALF+BAY group, F4/80 expression was reduced significantly (Figure 3(c)).

The expression of the M2 macrophage marker (CD163) in rat serum and liver tissues was detected, and it shows that CD163 was notably upregulated after adding JDHY or BAY compared with the ALF group (Figures 4(a)–4(c)). Meanwhile, expression of the anti-inflammatory factors IL-13 and IL-10 in serum and liver tissue of ALF rats was also upregulated, while expression of the M1 macrophages IL-1*β*, IL-6, IFN-*γ*, and TNF-*α* was declined (Figures 4(d) and 4(e)). All results indicated that JDHY could restore immunomodulation and could reduce M1 macrophage-caused inflammatory response in ALF rats.

### 3.4. JDHY Can Inhibit the Activation of the NF-*κ*B Signaling Pathway in Liver Tissue of Rats with Acute Liver Failure

As the NF-*κ*B pathway inhibitor BAY could significantly affect the immunoregulation and inflammatory response in rats with liver failure, a further study was conducted to investigate whether the treatment of ALF was associated with the NF-*κ*B signaling pathway. The result indicated that the ratio of p-IK*βα*/IK*βα*, p-IKK*β*/IKK*β*, and p-NF-*κ*B/NF-*κ*B was significantly increased in ALF rats, while JDHY could reduce their expression (Figure 5). All these suggested that the treatment of liver failure with JDHY might be associated with the inhibition of activating the NF-*κ*B signaling pathway.

## 4. Discussion

Liver failure, a serious liver damage brought by a series of factors, is also called hepatic failure. It leads to severe imbalance or decompensation of hepatic synthesis detoxification, biotransformation, excretion, and other functions [16]. Also, liver failure causes a variety of clinical syndromes such as coagulation disorders, jaundice, hepatic ascites, and encephalopathy [1]. The pathogenesis of liver failure is still unclear. The “two hits” hypothesis and “three hits” hypothesis are currently the most recognized theories. But whichever theory emphasizes the importance of immune impairment and inflammatory response in the development of liver failure. At present, more and more scholars agree with “Two-hit theory with immune-inflammatory injury as the core.” That is, on the basis of direct damage to liver cells such as HBV, through lipopolysaccharide- (LPS-) induced core pathogenesis of liver failure (endotoxin-macrophage-cytokine storm), an excessive and long-lasting immune-inflammatory response is produced. This response causes a “second hit” to the liver, ultimately resulting in the occurrence of liver failure [17, 18].

JDHY originated from Yinchenhao decoction in *Treatise on Febrile Diseases Caused by Cold* (a traditional Chinese medicine book written by Zhang Zhongjing). According to the etiopathology of “phlegm-stasis cementation” in ALF, JDHY has been refined by Professor Mao Dewen who comes from the First Affiliated Hospital of Guangxi University of Chinese Medicine. And the clinical treatment effect of JDHY has been confirmed. It can truncate the progression of liver failure, reduce the complications, ameliorate the prognosis, and enhance the survival rate [19]. However, there are few researches about influence and mechanism of JDHY on immune function of liver failure. In this research, D-GaIN/LPS was successfully applied to induce the ALF rat model, which mainly manifested liver function and coagulation function impairment. While the liver tissue injury was significantly improved in ALF rats pretreated with JDHY, further, JDHY could inhibit Bax and cleaved caspase-3 expression and promote Bcl-2 and PCNA expression in the liver cells of ALF rats. All results suggested that JDHY could inhibit the apoptosis and promote the proliferation of liver cells in ALF rats.

The pathogenesis of hepatitis B virus-associated acute-chronic liver failure (HBV-ACLF) was affected a lot by T cell-mediated immune damage. During HBV-ACLF, the diversity of the T cell repertoire was reduced significantly while the proportion of CD8+ T cells was upregulated notably [20]. This research also indicated that CD8+ T cells were significantly upregulated and CD4+ T cells were significantly decreased in ALF rats, while JDHY could downregulate the proportion of CD8+ T cells and upregulate CD4+ T cells.

Under the catalytic transport of the LPS-binding proteins, intestinal LPS binds to the TLR4-CD14-MD2 complex on the Kupffer cell surface to stimulate MyD88 and TRIF aggregation, thereby causing the activation of the NF-*κ*B signaling pathway. The activated Kupffer cells release large amounts of inflammatory factors including TNF-*α*, IL-1, IL-1, IL-10, IL-18, and reactive oxygen species (ROS). And these inflammatory factors act on the liver cell biofilms and damage the liver cells, thereby causing liver failure [21, 22]. Meanwhile, according to the study, interleukins IL-10 and IL-6 can upregulate CD163 expression in monocytes [23, 24]. Unlike cytokines, most proinflammatory factors such as IFN*γ*, LPS, and TNF-*α* can downregulate the expression of CD163 [25, 26].

CD163 is a specific M2 macrophage marker that plays an antioxidant role and regulates human immunity by removing free hemoglobin. SCD163 in plasma is shed from CD163 on the surface of membrane cells, which is thought to be able to inhibit T cell proliferation and regulate immunity [11, 27]. It has been confirmed that CD163/sCD163, as a marker of monocyte-macrophage activation, plays an antioxidant and anti-inflammatory role in liver failure. By animal experiments, some studies have speculated [10, 28] that endotoxemia promotes red blood cell destruction to increase and release large amounts of free hemoglobin under pathological conditions of acute liver failure; at this time, CD163 expression in macrophages is increased in liver tissue. With the deepening of research, it is increasingly recognized that the expression of CD163/sCD163 in liver failure can affect the innate immune response and control the development of adaptive immune response. And CD163/sCD163 is an important factor that takes part in and affects the core mechanism of “endotoxin → macrophage → cytokine storm.” In this study, we also found that JDHY could promote CD163 expression in the sCD163 of serum and liver tissues of ALF rats. Furthermore, JDHY increased the expression of IL-10 and IL-13 in serum and liver tissues of ALF rats, while the expression (IL-6, IL-1*β*, TNF-*α*, and IFN-*γ*) was decreased. The result indicated that JDHY could inhibit the inflammatory response caused by M1 macrophages. Further analysis of its molecular mechanism revealed that JDHY inhibited the phosphorylation expression of IKK*β*, IK*βα*, and NF-*κ*B in the liver tissues of ALF rats. The molecular mechanism of JDHY indicated that the protection of the liver of JDHY on ALF rats might be related to the inhibition of the activation of the NF-*κ*B pathway. This is consistent with Li et al. [29]; they have found that, by inhibiting the activity of NF-*κ*B, tumor necrosis factor *α*-induced protein 3 (A20) can inhibit D-GaIN/LPS-induced hepatocyte apoptosis in rats with ALF.

## 5. Conclusion

In summary, this study has found that JDHY can reduce liver injury, hepatocyte apoptosis, and inflammatory response, restore immune regulation, and promote liver cell proliferation in ALF rats. The mechanism of JDHY may be related to the inhibition of the NF-*κ*B signaling pathway in liver tissues. The results can provide reliable theoretical support for the clinical use of JDHY.

## Figures and Tables

**Figure 1:** JDHY can improve liver damage in ALF rats. (a–d) Biochemical tests were applied to check changes in indicators of liver function (AST, ALT, ALP, and TBiL) in serum of each group. In the ALF group (*n* = 10), the level of ALT, AST, ALP, and TBiL was higher compared with that in the control group (*n* = 6), while the level of AST, ALT, ALP, and TBiL was upregulated significantly in the ALF+JDHY group (*n* = 10) and ALF+BAY group (*n* = 10). (e, f) Biochemical tests were used to measure the prothrombin activity (PTA) of rats and the count of platelet (PLT). (g) Histopathological damage to the rat liver was checked by H&E staining. ^∗∗^*P* < 0.01 vs. control group (*n* = 6), ^##^*P* < 0.01 vs. ALF group (*n* = 10). BAY: NF-*κ*B inhibitor.

**Figure 2:** JDHY can decline liver apoptosis in ALF rats. (a) Western blot was used to check apoptosis-related protein expression (Bax, cleaved caspase-3, and Bcl-2) in rat liver tissues. Compared with the control group (*n* = 6), Bax expression and cleaved caspase-3 expression were notably increased in the liver tissues of the ALF group (*n* = 10) and Bcl-2 expression was significantly declined. While both Bax and cleaved caspase-3 expression were significantly declined in the liver tissues of ALF rats, Bcl-2 protein expression was significantly upregulated in the ALF+JDHY group (*n* = 10) and ALF+BAY group (*n* = 10). (b) Immunohistochemistry was utilized to determine PCNA expression in liver tissues of rats. It indicated that the positive expression of PCNA in the liver tissues of the ALF group was notably lower compared with that of the control group. Through the addition of JDHY and BAY, the level of PCNA was increased. ^∗∗^*P* < 0.01 vs. control group (*n* = 6), ^##^*P* < 0.01 vs. ALF group (*n* = 10).

**Figure 3:** Effects of JDHY on immune function in ALF rats. (a) Flow cytometry was utilized to check the proportion of CD4+ T cells in PBMCs of rats, CD4+ T cells in PBMCs were significantly reduced in the ALF group (*n* = 10), and CD4+ T cells were significantly upregulated in the ALF+JDHY group (*n* = 10) and ALF+BAY group (*n* = 10). (b) Flow cytometry was applied to determine the proportion of CD8+ T cells in PBMCs of rats; CD8+ T cells notably increased in the ALF group (*n* = 10) while they were notably reduced in the ALF+JDHY group (*n* = 10) and ALF+BAY group (*n* = 10). (c) Immunohistochemistry was used to measure F4/80 expression in rat liver tissues. ^∗∗^*P* < 0.01 vs. control group (*n* = 6), ^##^*P* < 0.01 vs. ALF group (*n* = 10).

**Figure 4:** Effect of JDHY on macrophages in ALF rats. (a) ELISA was applied to measure sCD163 expression in rat serum. (b) qRT-PCR was applied to determine CD163 expression in liver tissues of rats. (c) Western blot was adopted to measure CD163 expression in liver tissues of rats. (a)–(c) showed that the expression of CD163 was notably upregulated in the ALF+JDHY group (*n* = 10) and ALF+BAY group (*n* = 10) compared with the ALF group (*n* = 10). (d) ELISA was utilized to check the content of IL-10, IL-13, IL-1*β*, IL-6, IFN-*γ*, and TNF-*α* in rat serum. (e) qRT-PCR was adopted to check the expression of IL-1*β*, IL-10, IL-6, IL-13, TNF-*α*, and IFN-*γ*. ^∗∗^*P* < 0.01 vs. control group (*n* = 6), ^##^*P* < 0.01 vs. ALF group (*n* = 10).

**Figure 5:** Effect of JDHY on the NF-*κ*B signaling pathway in liver tissue of liver failure rats. Western blot was utilized to detect the expression of p-IKK*β*/IKK*β*, p-NF-*κ*B/NF-*κ*B, and p-IK*βα*/IK*βα* in liver tissue of rats in each group. It showed that the ratio of p-IK*βα*/IK*βα*, p-IKK*β*/IKK*β*, and p-NF-*κ*B/NF-*κ*B was significantly increased in the ALF group (*n* = 10), while JDHY (*n* = 10) could reduce their expression. ^∗∗^*P* < 0.01 vs. control group (*n* = 6), ^##^*P* < 0.01 vs. ALF group (*n* = 10).

**Table 1:** Primers and sequences.

Primers	Sequences (5′-3′)
IL-10	F: CGAGATGCCTTCAGCAGAG
	R: CGCCTTGATGTCTGGGTCTT

IL-6	F: ACTTCCATCCAGTTGCCTTCTTGG
	R: TTAAGCCTCCGACTTGTGAAGTGG

IL-13	F: GTCCCAGTGTAGCACCAATGA
	R: GCTCAGGTTGTGCCAAATGC

IL-1*β*	F: GTGGCTGTGGAGAAGCTGTGG
	R: CGGAGCCTGTAGTGCAGTTGTC

TNF-*α*	F: GATGGGTTGTACCTTGTCTACT
	R: CTTTCTCCTGGTATGAGATAGC

IFN-*γ*	F: CAGGCCATCAGCAACAACATAAGC
	R: AGCTGGTGGACCACTCGGATG

CD163	F: AGTCTGCTCAAGATACACAGAAA
	R: GGGGTAGAAAGGGCAACTCC

GAPDH	F: TCACCATCTTCCAGGAGCGAGAC
	R: AGACACCAGTAGACTCCACGACATAC

## Data Availability

The data used to support the findings of this study cannot be made freely available. Requests for access to these data should be made to Dewen Mao (maogw@gxtcmu.edu.cn).
